# Poor Prognosis in Low-Grade Endometrial Stromal Sarcoma With Cyclin-Dependent Kinase Inhibitor 2A Homozygous Deletion: A Case Study

**DOI:** 10.7759/cureus.54066

**Published:** 2024-02-12

**Authors:** Atsushi Mori, Kyosuke Kamijo, Megumi Sano, Tsutomu Muramoto, Yaeko Kobayashi

**Affiliations:** 1 Gynecology, Nagano Municipal Hospital, Nagano, JPN

**Keywords:** cyclin-dependent kinase inhibitor 2a, chemotherapy, hormone therapy, prognosis, low-grade endometrial stromal sarcoma

## Abstract

Low-grade endometrial stromal sarcoma (LGESS) typically has a favorable prognosis. Hormone therapy is considered the first choice of treatment for recurrent LGESS. In this report, we describe a case of recurrent LGESS where hormone therapy was ineffective, chemotherapy showed a partial response (PR), and pazopanib resulted in stable disease (SD). A 50-year-old patient with LGESS underwent a simple total hysterectomy and bilateral adnexectomy (pT1aN0M0, stage IA). Five years later, pelvic tumors and ascites were observed. Exploratory laparoscopy revealed bloody ascites, an 8 cm pelvic tumor, and extensive peritoneal dissemination. Nuclear atypia of the tumor cells was mild, pleomorphism and mitotic figures could not be confirmed, and necrosis was not observed. Immunostaining was positive for CD10 and estrogen receptor, negative for the BCL6 corepressor (BCOR), and showed a low Ki-67 index. Fluorescence in situ hybridization (FISH) examination of the tissue showed rearrangement of the JAZF zinc finger 1 (JAZF1) gene. Multigene panel testing revealed a homozygous deletion of cyclin-dependent kinase inhibitor 2A (CDKN2A). Accordingly, the patient was diagnosed with recurrent LGESS and was treated with an aromatase inhibitor, followed by medroxyprogesterone acetate; both were ineffective. The patient had a PR to chemotherapy (doxorubicin/ifosfamide) and SD to pazopanib. The patient died 1.5 years after recurrence. In conclusion, we present a case of LGESS with a poor prognosis where hormone therapy was ineffective, and chemotherapy and pazopanib were both partially effective. The poor prognosis may have been associated with the CDKN2A homozygous deletion.

## Introduction

Low-grade endometrial stromal sarcoma (LGESS) is a rare and indolent tumor with a generally favorable overall prognosis. The 5-year overall survival rate for stages I-II is approximately 90% [1]. LGESS is associated with a 10-20% recurrence risk, with characteristic late recurrences occurring after 10-30 years [2]. Recurrences can manifest locally in the vaginal or pelvic regions, and distant metastases may develop in areas such as the abdominal wall or lungs [3]. Hormone therapies, such as progesterone and letrozole, play a substantial role in managing recurrent LGESS [4]. Hormone therapy is effective in 80-90% of patients with recurrent LGESS, and this effect is long-lasting. Patients who respond well to hormone therapy tend to have a favorable prognosis [5-7]. However, specific criteria that could identify patients who would benefit from hormone therapy are yet to be established. In cases where hormone therapy proves ineffective, chemotherapy is considered, although the extent of its effectiveness remains uncertain.

Cyclin-dependent kinase inhibitor 2A (CDKN2A) is a tumor suppressor gene that encodes a protein responsible for inhibiting the activity of cyclin-dependent kinases 4/6. Alterations in CDKN2A have been described in a wide spectrum of cancer types, including familial melanoma [8], Burkitt's lymphoma [9], and esophageal squamous cell carcinoma [10].

In the current case report, we present a patient with recurrent LGESS who had a poor prognosis. The patient had an unsatisfactory response to hormone therapy and showed a partial response (PR) to chemotherapy, and stable disease (SD) to pazopanib. According to multigene panel testing, the patient had a homozygous deletion of CDKN2A. Homozygous CDKN2A deletion in LGESS may be associated with a poor prognosis.

## Case presentation

A 50-year-old woman, who had had two full-term vaginal deliveries and was known for osteoarthritis, presented to our hospital complaining of excessive menstrual bleeding. She was diagnosed with submucosal uterine fibroids. Subsequently, she underwent a total abdominal hysterectomy and bilateral adnexectomy. The pathological examination of the tissue sample revealed a 3 cm leiomyoma, and irregular islands of tumor cells permeating the myometrium without an associated stromal response. Histologically, the tumor cells resembled endometrial stromal cells with mild atypia (Figure 1). Immunohistochemical staining showed positivity for CD10 and estrogen receptor (ER), and focal positivity for cyclin D1. The postoperative pathological diagnosis was LGESS. The postoperative computed tomography (CT) revealed no lymph node enlargement or distant metastases. The clinical diagnosis was LGESS (stage IA).

**Figure 1:** Histological examination of the resected uterus. (A) Irregular nests of tumor cells permeate the myometrium without stromal reaction (x4 hematoxylin and eosin). (B) The tumor cells have uniform, oval to fusiform nuclei with no or minimal atypia and scant cytoplasm (x20 hematoxylin and eosin).

Five years later, she visited a gynecologist for abdominal distension. Magnetic resonance imaging (MRI) revealed gross ascites and an 8 cm mass in the lower abdomen (Figure 2).

**Figure 2:** Magnetic resonance imaging (MRI) at the time of recurrence. (A) Sagittal T2-weighted MRI reveals a pelvic mass in 8 cm diameter (arrow) and ascites. (B) Axial T2-weighted MRI.

Exploratory laparoscopy confirmed the ascites and revealed a lower abdominal mass, omental deposits, and extensive peritoneal dissemination (Figure 3).

**Figure 3:** First exploratory laparoscopic finding. (A) Extensive peritoneal dissemination is revealed. (B) Pelvic recurrent mass (arrow).

Tissue was collected from the peritoneal lesions for histological examination, which revealed short, spindle-shaped tumor cells with mild atypia and pleomorphism. Neither mitotic figures nor necrosis were observed (Figure 4A). Immunohistochemical staining was positive for CD10 and ER (Figures 4B, 4C) and focally positive for cyclin D1 (Figure 4D). The Ki-67 index was low (~5%). The pathological findings were similar to those of the LGESS found in the extracted uterus five years before.

**Figure 4:** Section from the metastatic tumor on the peritoneum. (A) The nuclei are small and round with mild atypia (x20 hematoxylin and eosin). (B) Positive immunohistochemical staining for CD10 (x20). (C) Positive immunohistochemical staining for estrogen receptor (x20). (D) Focally positive immunohistochemical staining for cyclin D1 (x20).

Fluorescence in situ hybridization (FISH) examination of the peritoneal deposits revealed a rearrangement of the JAZF zinc finger 1 (JAZF1) gene (Figure 5A). Immunohistochemical staining was negative for the BCL6 corepressor (BCOR) (Figure 5B). Multigene panel testing (OncoGuide™ NCC Oncopanel System) revealed a homozygous deletion of CDKN2A.

**Figure 5:** (A) Fluorescence in situ hybridization targeting JAZF1 gene. (B) Immunohistochemical staining for BCOR on metastatic tumor. (A) Fluorescence in situ hybridization (FISH) shows JAZF1 rearrangement using a dual color break-apart probe (arrows). (B) Immunohistochemical staining for BCOR is negative (x20).

Based on these findings, the tumor was diagnosed as recurrent LGESS. An aromatase inhibitor (letrozole 2.5 mg/day) was administered immediately for 30 days. Despite the administration of letrozole, the tumor rapidly increased in size, leading to a change in treatment from letrozole to medroxyprogesterone acetate (MPA 600 mg/day). While receiving MPA, symptoms such as abdominal distension and fatigue worsened. Therefore, it was decided to transition to chemotherapy before the overall condition deteriorated (Figure 6).

**Figure 6:** Clinical course and CT images (1) Computed tomography (CT) image before treatment. An arrow shows the recurrent tumor in the pelvis. The tumor size is 122 mm×41 mm. (2) CT image after hormone therapy. The tumor (arrow) has rapidly increased in size to 149 mm×79 mm despite hormone therapy. (3) CT image after the seventh cycle of doxorubicin/ifosfamide (DOX/IFM) therapy. The tumor has shrunk to 81 mm×52 mm. (4) CT image during the administration of pazopanib. The tumor size (70 mm×39 mm) has not changed. a: first exploratory laparoscopy  b: second exploratory laparoscopy

Because the hormone therapy was considered ineffective, seven cycles of a doxorubicin/ifosfamide (DOX 50 mg/m2, IFM 2 g/m2) regimen were administered. After the seventh cycle of chemotherapy, the tumor's long axis reduced from 149 mm to 81 mm, and the ascites markedly decreased. The effect was a partial response (PR) as per Response Evaluation Criteria in Solid Tumors v1.1. A second exploratory laparoscopy was performed. However, many peritoneal tumor deposits were observed. Since optimal cytoreduction was deemed unfeasible, cytoreduction surgery was not performed. This regimen was discontinued owing to IFM-induced renal dysfunction. Subsequently, pazopanib (800 mg/day) was administered for approximately 150 days. During this time, the tumor size, as well as the amount of ascites, showed little change, and the patient's condition remained stable (SD) (Figure 6). However, the tumor gradually became unresponsive to pazopanib therapy. The patient died of the disease 1.5 years after its recurrence.

## Discussion

LGESS is a rare and indolent tumor, and the overall prognosis is generally favorable. Among 310 cases with Stage I disease, 5-year overall survival was 100% for Stage IA (size <5cm) and 93% for Stage IB (>5 cm) [1]. For recurrent LGESS cases, therapy with progestins or aromatase inhibitors is recommended. One report showed that nine of 11 patients with recurrent LGESS treated with hormonal therapy had a complete or partial response [5]. Another report showed that four of five patients with recurrent LGESS responded to letrozole treatment [6]. Hormonal agents have been reported to be effective over the long term in many studies. Second-line hormonal therapy has proven effective even in cases that progress after first-line endocrine treatment. For cases still progressing after hormonal therapy, chemotherapy with doxorubicin-based regimens or gemcitabine plus docetaxel is employed. Surgery may be chosen only if optimal cytoreduction is achievable. In cases of unresectable localized recurrence, consideration may also be given to radiation therapy [1]. Regarding pazopanib, a study has indicated it as a treatment option for metastatic soft tissue sarcoma following chemotherapy [11]. However, there are few reported cases of pazopanib use for ESS.

The histopathological characteristic of LGESS involves proliferative-phase endometrial stromal-type tumor cells permeating the myometrium, with or without lymphovascular invasion. The tumor cells have uniform, oval to fusiform nuclei with no or minimal atypia and scant cytoplasm. LGESS exhibits diffuse positivity for CD10, ER, and PR immunohistochemistry, focal positivity for cyclin D1, and negative or focal positivity for BCOR [12,13]. In recent years, genetic testing has played an essential role in diagnosing ESS. The representative gene abnormality of LGESS is the JAZF1-SUZ12 fusion gene; however, other fusion genes include PHA-JAZF1, EPC1-PHF1, and MEAF6-PHF1.

The tumor cells in the present case were short and spindle-shaped and had a slightly high nuclear/cytoplasmic ratio; however, severe nuclear atypia, pleomorphism, mitosis, and necrosis were not observed. Immunohistochemical staining was positive for CD10 and ER and focally positive for cyclin D1. FISH confirmed the presence of the JAZF1 fusion gene. The partner gene could not be identified; however, additional immunostaining for BCOR was negative. Based on these results, the tumor was diagnosed as recurrent LGESS with the JAZF1 fusion gene.

The CDKN2A locus encodes p16INK4A and p14ARF. These proteins play critical roles in the suppression of cancer cells. CDKN2A/B mutations or deletions have been observed in several types of cancer. Cases of ESS with CDKN2A/B deletion showing BCOR internal tandem duplication or various BCOR/BCORL1 rearrangements have been reported [14]. Using comprehensive genomic profiling, Lin et al. examined 31 ESS genes and found that 28% of cases had a CDKN2A homozygous deletion [15]. CDKN2A/B homozygous deletion has also been reported in a case of recurrent LGESS with the JAZF1-BCORL1 fusion gene [16]. CDKN2A homozygous deletions have been reported to be associated with prognosis in various cancer types. A study reported CDKN2 homozygous deletion in 18% of ovarian cancer cases, which is associated with poor prognosis [17]. Other studies have reported that CDKN2A homozygous deletion is associated with prognosis in cases of malignant IDH (isocitrate dehydrogenase)-mutant gliomas [18], and pleural mesothelioma [19]. Kommoss reported p16 being a prognostic marker in HGESS with the YWHAE::NUTM2 gene fusion [20]. Based on these reports, the poor prognosis in this case may be related to CDKN2A homozygous deletion.

## Conclusions

Low-grade endometrial stromal sarcoma (LGESS) is a rare and indolent tumor with a generally favorable overall prognosis. For patients with recurrent LGESS, hormone therapy is the preferred first treatment of choice. However, the definitive effectiveness of chemotherapy or pazopanib for recurrent disease remains unclear. In the current case report, we present a patient with recurrent LGESS who had a poor prognosis. The patient had an unsatisfactory response to hormone therapy and showed a partial response (PR) to chemotherapy, and stable disease (SD) to pazopanib. The poor prognosis is possibly associated with the CDKN2A homozygous deletion.

## References

[1] Gadducci A, Multinu F, De Vitis LA, Cosio S, Carinelli S, Aletti GD (2023). Endometrial stromal tumors of the uterus: Epidemiology, pathological and biological features, treatment options and clinical outcomes. Gynecol Oncol.

[2] Thiel FC, Halmen S (2018). Low-grade endometrial stromal sarcoma - a review. Oncol Res Treat.

[3] Bai H, Yang J, Cao D (2014). Ovary and uterus-sparing procedures for low-grade endometrial stromal sarcoma: a retrospective study of 153 cases. Gynecol Oncol.

[4] (2024). NCCN guidelines version 1.2024 uterine neoplasms. https://www.nccn.org/guidelines/guidelines-detail?category=1&id=1473&utm_medium=email&utm_source=transaction.

[5] Dahhan T, Fons G, Buist MR, Ten Kate FJ, van der Velden J (2009). The efficacy of hormonal treatment for residual or recurrent low-grade endometrial stromal sarcoma. A retrospective study. Eur J Obstet Gynecol Reprod Biol.

[6] Pink D, Lindner T, Mrozek A, Kretzschmar A, Thuss-Patience PC, Dörken B, Reichardt P (2006). Harm or benefit of hormonal treatment in metastatic low-grade endometrial stromal sarcoma: single center experience with 10 cases and review of the literature. Gynecol Oncol.

[7] Gadducci A, Cosio S, Romanini A, Genazzani AR (2008). The management of patients with uterine sarcoma: a debated clinical challenge. Crit Rev Oncol Hematol.

[8] Aoude LG, Wadt KA, Pritchard AL, Hayward NK (2015). Genetics of familial melanoma: 20 years after CDKN2A. Pigment Cell Melanoma Res.

[9] Robaina MC, Faccion RS, Arruda VO (2015). Quantitative analysis of CDKN2A methylation, mRNA, and p16(INK4a) protein expression in children and adolescents with Burkitt lymphoma: biological and clinical implications. Leuk Res.

[10] Qureshi MA, Jan N, Dar NA, Hussain M, Andrabi KI (2012). A novel p16(INK4A) mutation associated with esophageal squamous cell carcinoma in a high risk population. Biomarkers.

[11] van der Graaf WT, Blay JY, Chawla SP (2012). Pazopanib for metastatic soft-tissue sarcoma (PALETTE): a randomised, double-blind, placebo-controlled phase 3 trial. Lancet.

[12] Chiang S, Lee CH, Stewart CJ (2017). BCOR is a robust diagnostic immunohistochemical marker of genetically diverse high-grade endometrial stromal sarcoma, including tumors exhibiting variant morphology. Mod Pathol.

[13] Denschlag D, Ackermann S, Battista MJ (2019). Sarcoma of the uterus. Guideline of the DGGG and OEGGG (S2K level, AWMF Register Number 015/074, February 2019). Geburtshilfe Frauenheilkd.

[14] Kommoss FK, Chiang S, Köbel M (2022). Endometrial stromal sarcomas with BCOR internal tandem duplication and variant BCOR/BCORL1 rearrangements resemble high-grade endometrial stromal sarcomas with recurrent CDK4 pathway alterations and MDM2 amplifications. Am J Surg Pathol.

[15] Lin DI, Hemmerich A, Edgerly C (2020). Genomic profiling of BCOR-rearranged uterine sarcomas reveals novel gene fusion partners, frequent CDK4 amplification and CDKN2A loss. Gynecol Oncol.

[16] Allen AJ, Ali SM, Gowen K, Elvin JA, Pejovic T (2017). A recurrent endometrial stromal sarcoma harbors the novel fusion JAZF1-BCORL1. Gynecol Oncol Rep.

[17] Kudoh K, Ichikawa Y, Yoshida S (2002). Inactivation of p16/CDKN2 and p15/MTS2 is associated with prognosis and response to chemotherapy in ovarian cancer. Int J Cancer.

[18] Appay R, Dehais C, Maurage CA (2019). CDKN2A homozygous deletion is a strong adverse prognosis factor in diffuse malignant IDH-mutant gliomas. Neuro Oncol.

[19] Kobayashi N, Toyooka S, Yanai H (2008). Frequent p16 inactivation by homozygous deletion or methylation is associated with a poor prognosis in Japanese patients with pleural mesothelioma. Lung Cancer.

[20] Kommoss FK, Mar LM, Howitt BE (2023). High-grade endometrial stromal sarcomas with YWHAE::NUTM2 gene fusion exhibit recurrent CDKN2A alterations and absence of p16 staining is a poor prognostic marker. Mod Pathol.

